This article has been retracted.

# Sagunja-Tang Improves Lipid Related Disease in a Postmenopausal Rat Model and HepG2 Cells

**DOI:** 10.1155/2015/321407

**Published:** 2015-04-22

**Authors:** Hiroe Go, Jin Ah Ryuk, Hye Won Lee, In Sil Park, Ki-Jung Kil, Sunmin Park, Dong il Kim, Byoung Seob Ko

**Affiliations:** ^1^Korean Medicine Convergence Research Division, Korea Institute of Oriental Medicine, 1672 Yuseongdae-ro, Yuseong-gu, Daejeon 305-811, Republic of Korea; ^2^College of Oriental Medicine, Joongbu University, 201 Daehak-Ro, Chubu-Myeon, Geumsan-Gun, ChungNam 312-702, Republic of Korea; ^3^Food and Nutrition, Obesity/Diabetes Center, Hoseo University, 165 Sechul-Ri, Bae Bang-Yup, Asan-Si, Chungcheongnam-do 336-795, Republic of Korea; ^4^Dongguk University Ilsan Oriental Hospital, 27 Dongguk-Ro, Ilsandong-Gu, Goyang-Si, Gyeonggi-Do 410-773, Republic of Korea

## Abstract

The present study was conducted to investigate the effect of Sagunja-tang on the lipid related disease in a rat model of menopausal hyperlipidemia and lipid accumulation in methyl-*β*-cyclodextrin-induced HepG2 cells. In *in vivo* study using menopausal hyperlipidemia rats, Sagunja-tang reduced retroperitoneal and perirenal fat, serum lipids, atherogenic index, cardiac risk factor, media thickness, and nonalcoholic steatohepatitis score, when compared to menopausal hyperlipidemia control rats. In HepG2 cells, Sagunja-tang significantly decreased the lipid accumulation, total cholesterol levels, and low-density/very-low-density lipoprotein levels. Moreover, Sagunja-tang reversed the methyl-*β*-cyclodextrin-induced decrease in the protein levels of critical molecule involved in cholesterol synthesis, sterol regulatory element binding protein-2, and low-density lipoprotein receptor and inhibited protein levels of 3-hydroxy-3-methylglutaryl coenzyme A reductase as well as activity. Phosphorylation level of AMP-activated protein kinase was stimulated by Sagunja-tang. These results suggest that Sagunja-tang has effect on inhibiting hepatic lipid accumulation through regulation of cholesterol synthesis and AMPK activity *in vitro*. These observations support the idea that Sagunja-tang is bioavailable both *in vivo* and *in vitro* and could be developed as a preventive and therapeutic agent of hyperlipidemia in postmenopausal females.

## 1. Introduction

Hyperlipidemia is defined as elevated lipid levels in the blood, including cholesterol, cholesterol esters, phospholipids, and triglycerides. Cholesterol is a naturally occurring fat or lipid that is present in the blood and other cells in the body. Cholesterol is produced by the body itself and is also obtained from dietary animal food sources. Cholesterol is transported in the blood as large lipoproteins, including high-density lipoproteins (HDLs) and low-density lipoproteins (LDLs). Cholesterol is necessary for proper body functioning and functions to protect health, including cardiovascular health. However, the presence of excessive amounts of total cholesterol results in the ability of cholesterol to adhere to artery walls as plaques. Cholesterol plaque formation prevents proper blood flow through the arteries and leads to an increased risk for developing cardiovascular diseases, including atherosclerosis, heart disease, blood clots, hypertension, heart attack, and stroke [1]. Moreover, hyperlipidemia also induces fatty liver diseases, including nonalcoholic fatty liver disease (NAFLD) and nonalcoholic steatohepatitis (NASH) [2]. The management of hyperlipidemia is associated with reduced risks for these diseases.

Postmenopausal females are at higher risk than age-matched premenopausal females for a number of health conditions, such as hyperlipidemia, cardiovascular disease, arteriosclerosis, and NASH, suggesting that menopause itself is a risk factor [3–5]. These conditions can be improved by hormone replacement therapy (HRT) or estrogen administration [4, 6]. However, HRT and estrogen replacement therapy (ERT) cause a small increase in the risk of developing serious diseases, such as breast cancer [7]. Therefore, the development of a safe, effective method of treating or preventing these diseases is urgently needed. In Asian countries, menopausal symptoms are understood as deficiencies in kidney and stomach/spleen energies and commonly treated successfully with herbal medicines.

Sagunja-tang (SGJT), a traditional Chinese remedy, consists of four oriental herbs (*Panax ginseng* C. A. Meyer,* Poria cocos* Wolf,* Atractylodes japonica* Koidzumi, and* Glycyrrhiza uralensis* Fischer) and has been used as a medicine to enhance vital energy and tonify the function of spleen and stomach in oriental countries. Therefore, SGJT is used for patients with reduced physical strength, a weakened immune system, and gastrointestinal diseases [8]. According to recent studies, SGJT exhibits several effects, such as antioxidant, anticancer, and immune stimulatory activity, radioprotective effects, and soothing effects [9–13]. Moreover, SGJT improves hyperlipidemia-induced high cholesterol in rabbits and also exhibits effects on uterine and ovarian function in the ovariectomized (OVX) postmenopausal rat model [14, 15]. Therefore, we hypothesized that SGJT affects lipid related diseases induced by a high-fat, high-cholesterol diet in the OVX postmenopausal rat model.

Cholesterol is synthesized and utilized via tightly regulated system mediated by sterol regulatory element binding protein 2 (SREBP2) [16, 17]. SREBP2 regulates cholesterol metabolism primarily through the regulation of genes associated with cholesterol uptake and synthesis, such as low-density lipoprotein receptor (LDLR) and 3-hydroxy-3-methylglutaryl coenzyme A reductase (HMGCR) [18–20].

AMPK is a phylogenetically conserved serine/threonine protein kinase that is activated in response to a rising intracellular AMP : ATP ratio following ATP depletion [21]. Therefore, AMPK is considered a metabolic master switch, mediating cellular adaptation to the environment or nutritional stress factors [22]. Once activated, AMPK leads to concomitant inhibition of anabolic pathways such as cholesterol, fatty acid, and triglyceride synthesis, as well as to stimulation of fatty acid oxidation and ketogenesis [21, 23, 24].

The objective of this study was to evaluate the impact of SGJT on lipid related diseases induced by a high-fat, high-cholesterol diet in OVX rats. An additional aim was to investigate the effects and cellular mechanisms of SGJT on hepatic lipid accumulation in HepG2 hepatocellular carcinoma.

## 2. Materials and Methods

### 2.1. SGJT Preparation

The formula of SGJT consist of 4 herbs, including* Panax ginseng* C. A. Meyer (125 g),* Poria cocos* Wolf (125 g),* Atractylodes japonica* Koidzumi (125 g), and* Glycyrrhiza uralensis* Fischer (125 g). Briefly, 500.0 g of the 4 herb mixture was mixed and extracted by heating for 2 h in a 10-fold volume of water using an S-20,000 extractor (Sak IK Medical Company). After lyophilization, the resulting SGJT powder (113.8 g, yield: 22.76%) was collected and stored at 4°C until use. The SGJT extract (KIOM PH 130001) was stored at Korea Institute of Oriental Medicine (KIOM, Daejeon, Korea) until being used in this experiment.

### 2.2. Chromatographic Conditions of HPLC-Diode Array Detector (DAD)

For quantitative analysis, five of the reference compounds solutions, glycyrrhizin and liquiritin (1,000 *μ*g/mL), were prepared in 100% methanol and stored at 4°C. The standard solutions were prepared by six concentrations of diluted solutions (methanol). All calibration curves were attained by assessing the peak areas at six concentrations in the range of 10–500 *μ*g/mL for all reference compounds. The linearity of the peak area (*y*) versus concentration (*x*, *μ*g/mL) curve for each component was used to calculate the contents of the main Sagunja-tang. 102.8 mg of Sagunja-tang extract powder was subsequently resuspended in 10 mL distilled water for high-performance liquid chromatography (HPLC) analysis.

The contents of glycyrrhizin and liquiritin in the SGJT water extract were analyzed using a 1100 series HPLC instrument (Agilent Technologies, USA) with a Gemini C18 column (4.6 × 250 mm, 5 *μ*m; Phenomenex, USA). The mobile phase consisted of the solvents, distilled water (A) and acetonitrile with 0.1% formic acid (B). The following gradient was used: 0 min, A : B 80 : 20 (v/v); 10 min, A : B 60 : 40; 15 min, A : B 40 : 60; 30 min, A : B 15 : 85; and 40 min, A : B 0 : 100. The mobile phase flow rate was 1.0 mL/min, the column temperature was 30°C, the injection volume was 10 uL, and UV detection was at 254 nm (glycyrrhizin) and 280 nm (liquiritin).

### 2.3. Cell Culture and Treatment

HepG2 human hepatocellular carcinoma cells were purchased from the Korean Cell Line Bank (Seoul, Korea). HepG2 cells were cultured in DMEM supplemented with 10% fetal bovine serum, 100 U/mL penicillin, and 100 mg/mL streptomycin and maintained in a humidified incubator at 37°C under an atmosphere of 5% CO_2_. To induce cholesterol production, HepG2 cells were exposed to M*β*CD mixed with palmitic acid. When cells reached 70% confluence, they were incubated in 0.2% BSA-DMEM containing 20 *μ*g/mL M*β*CD, along with 30 *μ*M simvastatin or various concentrations (250–1,000 *μ*g/mL) of SGJT for 8 h.

### 2.4. Animals and Treatment

All experimental protocols and animal maintenance procedures used in this study were treated in accordance with the Guide for Care and Use of Laboratory Animals by the Institutional Animal Care and Use Committee (IACUC) of Korea Institute of Oriental Medicine (KIOM). Six-week-old female Sprague-Dawley rats (weight 225 ± 25 g) were obtained from Samtako (Osan-si, Korea) and maintained under a regular 12:12 h light:dark cycle at a controlled temperature (24 ± 2°C) and relative humidity (50–55%) in the Laboratory Animals Center at KIOM (Approval Number 13-026). After 1 week of acclimation, the rats underwent ovariectomy (*n* = 25) or sham operation (*n* = 5) under anesthesia by intramuscular injection of Zoletil and Rompun mixture. One week after the surgery, twenty-five OVX rats were randomly divided into three groups: (1) high-fat (45%), high-cholesterol (1%) diet (OVX-Con) (*n* = 5), (2) high-fat (45%), high-cholesterol (1%) diet with simvastatin (OVX-SV; 20 mg/kg) (*n* = 5), and (3) high-fat (45%), high-cholesterol (1%) diet with SGJT (OVX-SGJT; 50, 150, and 450 mg/kg) (*n* = 5 per each dose). Five sham-operated rats were assigned to a high-fat (45%), high-cholesterol (1%) diet (Sham). Simvastatin and SGJT were dissolved in phosphate-buffered saline (PBS) for daily oral administration. After eight weeks, rats were sacrificed under anesthesia and blood was collected for the estimation of total-cholesterol (TC), triglycerides (TG), high-density lipoprotein cholesterol (HDL), low-density lipoprotein cholesterol (LDL), atherogenic index, and cardiac risk factor. Liver tissue, retroperitoneal fat, perirenal fat, and arterial tissue were also collected.

### 2.5. Lipid Parameters

Serum TC, TG, and HDL levels were measured using a BS220 instrument (Mindray, Shenzhen, China). LDL levels were determined using the following equation: LDL = TC – HDL − (TG/5). TC and LDL/VLDL contents in HepG2 cells were determined using HDL and LDL/VLDL cholesterol assay kit according to the manufacturer's instructions. Briefly, HepG2 cells were seeded at a density of 1 × 10^5^ cells/well in 24-well plates and treated with 30 *μ*M simvastatin and various concentrations of SGJT (250–1000 *μ*g/mL) with M*β*CD in 0.2% BSA-DMEM for 8 h. Then cellular lipids were extracted with chloroform : isopropanol : NP-40 (7 : 11 : 0.1) in a microhomogenizer. Extracts were then centrifuged for 10 min at 15,000 g. Next, supernatants were transfer to a new tube, air dried at 50°C to remove chloroform, and placed under a vacuum for 30 min to remove any trace organic solvent. Dried lipids were then resuspended in 200 *μ*L cholesterol assay buffer by vortexing until homogeneous. TC and LDL/VLDL levels were assayed by measuring absorbance at 570 nm using a spectrophotometer.

### 2.6. Atherogenic Index and Cardiac Risk Factor

Atherogenic index and cardiac risk factor were determined using the following equations: atherogenic index = (TC − HDL)/HDL; cardiac risk factor = TC/HDL.

### 2.7. Histology

Rat livers were fixed with 4% neutral buffered formalin (NBF) and embedded in paraffin. Four-micron sections were then cut and stained with Hematoxylin and Eosin (H&E) to determine NASH scores. A diagnosis of NASH was established by the presence of a characteristic pattern of steatosis, lobular inflammation, and hepatocellular ballooning. Total scores of each component were then added to determine the presence or absence of NASH, with score ≥5 diagnosed as NASH and scores ≤2 defined as not NASH.

To measure retroperitoneal and perirenal fat accumulation, lipid tissues were fixed with 10% NBF and embedded in paraffin. Twenty-micron sections were then cut and stained with H&E and examined by light microscopy.

### 2.8. Cytotoxicity

The cell viability was examined by (4-[3-(4-iodophenyl)-2-(4-nitrophenyl)-2*H*-5-tetrazolio]-1,3-benzene disulfonate) (WST) assay. Briefly, HepG2 cells were seeded at a density of 2 × 10^4^ cells/well in 96-well plates and treated with 30 *μ*M simvastatin and various concentrations of SGJT (250–1,000 *μ*g/mL) with or without M*β*CD in 0.2% BSA-DMEM for 8 h. Then WST solution was added to each well and the cells were cultured for another 2 h, after which the optical density was read at 490 nm.

### 2.9. Oil Red O Staining

To measure total intracellular lipid content, HepG2 cells were stained using the Oil Red O method. Briefly, HepG2 cells were seeded at a density of 1 × 10^5^ cells/well in 24-well plates and treated with 30 *μ*M simvastatin and various concentrations of SGJT (250–1,000 *μ*g/mL) with or without M*β*CD in 0.2% BSA-DMEM for 8 h. Then cells were washed three times with PBS and fixed with 10% formalin for 10 min. After fixation, cells were washed with PBS and 60% isopropanol and stained for 1 h in a freshly diluted Oil Red O solution (stock solution, 3 mg/mL in isopropanol; working solution, 60% Oil Red O stock solution diluted in water). After staining, cells were washed with 60% isopropanol and PBS and photographed. For quantitative analysis of cellular lipids, isopropanol was added, followed by shaking at room temperature for 10 min. The extracted dye was removed by gentle pipetting and its absorbance at 500 nm was monitored using a spectrophotometer.

### 2.10. HMG-CoA Reductase Activity

Cells were cultured to 80% confluence at 37°C, incubated in 0.2% BSA-DMEM containing 20 *μ*g/mL M*β*CD, and treated with 30 *μ*M simvastatin or various concentrations of SGT (250 and 500 *μ*g/mL) for 8 h. Cells were then lysed in RIPA buffer (50 mM Tris-HCl [pH 7.4], 150 mM NaCl, 1.0% (v/v) NP-40, 0.5% (w/v) sodium deoxycholate, 1.0 mM EDTA, 0.1% (w/v) SDS, and 0.01% (w/v) sodium azide) containing protease inhibitors (Biocyc GmbH & Co. KG). HMG-CoA reductase activity was then determined using an HMG-CoA reductase assay kit, according to the manufacturer's instructions.

### 2.11. Western Blotting

Cells were cultured to 80% confluence at 37°C, incubated in 0.2% BSA-DMEM containing 20 *μ*g/mL M*β*CD, and treated with 30 *μ*M simvastatin or various concentrations of SGJT (250 and 500 *μ*g/mL) for 8 h. Cells were then lysed in RIPA buffer containing protease inhibitors. Lysates were incubated at 4°C for 30 min and then centrifuged at 14,000 rpm for 15 min at 4°C to remove detergent-insoluble material.

Protein concentration was determined using a Bio-Rad protein assay. Protein extracts (30–90 *μ*g) were then separated on 4–15% Mini-Protean TGX Precast Gels and transferred to a polyvinylidene fluoride membrane. The membranes were blocked with 1% bovine serum albumin in PBS-T (137 mM NaCl, 2.7 mM KCl, 4.3 mM Na_2_HPO_4_, 1.4 mM KH_2_PO_4_, and 0.1% Tween 20) and then incubated with the following antibodies: anti-HMGCR (C-1; 1 : 1,000), anti-SREBP2 (1C6; 1 : 1,000), anti-*β*-actin (C4; 1 : 1,000), anti-phospho-AMPK*α* (Thr172; 1 : 1,000), anti-AMPK*α* (1 : 1,000), and anti-LDL Receptor (1 : 1,000) antibodies. Membranes were then incubated overnight at 4°C with gentle shaking. Secondary antibodies included HRP-conjugated goat anti-mouse, goat anti-rabbit, and donkey anti-goat (1 : 10,000) antibodies, as appropriate. Antibody-bound proteins were visualized using an Immun-Star WesternC kit.

### 2.12. Statistical Analyses

All of the experiments were performed in triplicate and repeated at least three times. Data are expressed as a mean ± standard deviation. Statistical analysis was performed using the SPSS software version 12.0 (SPSS Inc., Chicago, IL) and data were evaluated for statistical significance using one-way ANOVA followed by Duncan's test (*P* < 0.05). The OVX and Sham groups and control and M*β*CD groups were compared using two-sample *t*-tests (*P* < 0.05).

## 3. Results

### 3.1. HPLC Analysis of Reference Compounds in SGJT

The reference standards of calibration curves for the glycyrrhizin and liquiritin were *y* = 6.2359*x* + 2.6833 (*R* ^2^ 0.998) and *y* = 15.9401*x* − 63.1150 (*R* ^2^ 0.999), respectively. HPLC analysis of SGJT and reference standard mixtures was carried out at 254 and 280 nm. The retention time of each compound was 12.89 min (liquiritin) and 27.83 min (glycyrrhizin). The contents of each component in SGJT aqueous extract were liquiritin 4.72 ± 0.056 mg/g and glycyrrhizin 17.49 ± 0.452 mg/g, respectively (Figure 1).

### 3.2. SGJT Affects the Body Weight and Abdominal Fat Accumulation of Menopausal Hyperlipidemic Rats Fed a High-Fat, High-Cholesterol Diet

We established a rat model of menopausal hyperlipidemia using OVX rats fed a high-fat, high-cholesterol diet. After 8 weeks, the body weights of all rats were measured (Table 1); the rats in the OVX group (OVX-Con) weighed more than those in the Sham group (Sham). In the SGT-treated groups (OVX-SGJT 50, 150, and 450), SGJT inhibited the OVX-induced weight gain. All rats were sacrificed at week 8, and the liver weights of each group were compared (Table 1). Although significantly increased liver weights were observed in the OVX-Con group compared with the Sham group, no significant differences were evident in the OVX-SV and OVX-SGJT groups relative to the OVX-Con group.

Overall fat volumes were also examined in retroperitoneal and perirenal fat deposits (Figure 2(a) and Table 1). The OVX-Con group significantly increased both retroperitoneal and perirenal fat volumes compared with the Sham group. All OVX-SGJT groups exhibited decreased retroperitoneal fat volumes and decreased perirenal fat volumes that were similar to those of the OVX-SV group.

### 3.3. SGJT Affects Serum Lipids in Menopausal Hyperlipidemic Rats Fed a High-Fat, High-Cholesterol Diet

The OVX-Con group exhibited significantly increased TC, TG, and LDL levels compared with the Sham group (Table 2). In contrast, HDL levels were decreased in the OVX-Con group compared with the Sham group (Table 2). The OVX-SV group and OVX-SGT groups decreased the OVX-induced changes in TC and LDL levels. TG levels were altered, but not significantly, in the OVX-SV and OVX-SGJT groups. The OVX-SV group and OVX-SGJT groups exhibited increased HDL levels relative to the OVX-Con group (Table 2).

### 3.4. SGJT Decreases the Risk of Arterial Sclerosis in Menopausal Hyperlipidemic Rats Fed a High-Fat, High-Cholesterol Diet

Arterial sclerosis is a medical condition in which an arterial wall stiffens as a result of fat accumulation. Increased levels of total plasma cholesterol and obesity represent significant risk factors for atherosclerosis and increased rates of cardiovascular death [25, 26]. As SGJT decreased the levels of fat accumulation in retroperitoneal and perirenal spaces and serum cholesterol levels in menopausal hyperlipidemic rats (Tables 1 and 2, Figure 2(a)), we next examined the effect of SGJT on the risk of arterial sclerosis by measuring the atherogenic index, cardiac risk factors, lumen diameter, and intima-media thickness (Table 3). The OVX-Con group exhibited significantly increased atherogenic index and cardiac risk factor scores compared to the Sham group. The OVX-SV and all OVX-SGJT groups exhibited lower atherogenic index and cardiac risk factor scores relative to the OVX-Con group (Table 3). Lumen diameter and intima-media thickness were also determined. The OVX-Con group had a lower overall lumen diameter than the Sham group. In contrast, the OVX-SGJT groups had a higher overall lumen diameter. In contrast, the OVX-Con group had increased intima-media thickness relative to the Sham group (Table 3). All OVX-SGJT groups had a decreased intima-media thickness, similar to that of the OVX-SV group (Table 3).

### 3.5. SGJT Ameliorates Hepatic Steatosis of Menopausal Hyperlipidemic Rats Fed a High-Fat, High-Cholesterol Diet

Obesity, diabetes, and hyperlipidemia are important risk factors for NASH; patients with fatty liver disease or an excessive accumulation of fat in liver hepatocytes are more likely to develop NASH [2, 27]. NASH is characterized by the presence of steatosis, lobular inflammation, and hepatocellular ballooning [28]. To determine the effect of SGJT on NASH development, rats were examined for the presence of major NASH symptoms, including steatosis, lobular inflammation, and hepatocellular ballooning. Although a greater number of fat vacuoles were observed in the OVX-Con group compared to the Sham group, both the OVX-SV and OVX-SGJT groups had fat accumulation levels similar to those of the Sham group (Figure 2(b)). Moreover, the scores of each NASH component (steatosis, lobular inflammation, and hepatocellular ballooning) were higher in the OVX-Con group relative to the Sham group. In the OVX-SV and OVX-SGJT groups, the scores of each NASH component were lower relative to the controls (Table 4).

### 3.6. SGJT Does Not Affect Viability of HepG2 Cells

Since SGJT showed improvement effects on hepatic steatosis* in vivo*, the effect and cellular mechanisms of SGJT on the hepatic lipid accumulation in HepG2 hepatocellular carcinoma were examined. We induced steatosis by M*β*CD. A WST assay was performed to evaluate the cytotoxicity of M*β*CD, SGJT, and simvastatin on the viability of HepG2 cells. As shown in Figure 3(a), increasing concentrations of SGJT (250–1,000 *μ*g/mL) exhibited no cytotoxic effects. Treatment of HepG2 cells with M*β*CD only resulted in a slight inhibition of cell growth (Figure 3(b)). M*β*CD added to cells pretreated with SGJT (250–1,000 *μ*g/mL) or simvastatin (30 *μ*M) was found to be nontoxic at the concentrations tested (Figure 3(b)).

### 3.7. SGJT Inhibits HepG2 Cellular Lipid Accumulation

To evaluate the inhibitory effects of SGJT on M*β*CD-induced lipid accumulation, HepG2 cells were treated with various concentrations of SGJT for 8 h; pretreatment with simvastatin was used as the positive control. Then, cells were stained with Oil Red O and quantified by measuring the absorbance at 500 nm. A significant increase in lipid deposition was observed in HepG2 cells treated with M*β*CD; however, this effect was attenuated in SGJT and simvastatin-treated cells (Figure 4(a)). This suggested that SGJT significantly inhibited M*β*CD-induced intracellular lipid accumulation in HepG2 cells. This result was confirmed by the quantification of TC and LDL/VLDL levels (Figures 4(b) and 4(c)). SGJT treatment significantly inhibited total cholesterol levels at all concentrations tested, and LDL/VLDL levels were also lower in these cells (Figure 4(c)).

### 3.8. SGJT Affects Cholesterol Synthesis in HepG2 Cells

Having established a direct link between SGJT and cholesterol synthesis, we sought to identify the mechanisms underlying this effect. Cholesterol homeostasis is tightly regulated by the transcription factor SREBP2 [17], which directly regulates the transcription of important genes involved in cholesterol synthesis, such as HMGCR and LDLR. We first investigated the effect of SGJT on HMGCR activity in HepG2 cells; SGJT decreased the activity of HMGCR relative to the controls (Figure 5(a)).

In addition to enzyme activity, we evaluated the effects of SGJT on the SREBP2, HMGCR, and LDLR levels in HepG2 cells. LDLR and SREBP2 protein levels were diminished in M*β*CD-treated cells but could be rescued to near wild-type levels by SGJT treatment (Figure 5(b)). In contrast, HMGCR protein levels were diminished by treatment with M*β*CD or SGJT (Figure 5(b)). These results show that SGJT attenuated lipid accumulation via the regulation of the genes involved in cholesterol synthesis.

### 3.9. SGJT Induces AMPK Phosphorylation in HepG2 Cells

AMPK is thought to act as a metabolic master switch in response to changes in cellular energy and plays a crucial role in regulating fat metabolism in the liver [29, 30]. Therefore, AMPK phosphorylation is used as a marker of AMPK activity. SGJT significantly increased AMPK phosphorylation compared with M*β*CD alone (Figure 6), suggesting that SGJT attenuated hepatic lipid accumulation through AMPK activation.

## 4. Discussion

Menopause is known to be associated with an increased incidence of metabolic syndrome and a variety of conditions (including dyslipidemia, insulin resistance, and obesity) that lead to an increased risk of cardiovascular disease, type 2 diabetes, NASH, and atherosclerosis [31]. Estrogen treatment reverses the effects of menopause on these diseases [32–34]. However, estrogen replacement therapy increases the risk of various cancers, including endometrial, breast, and ovarian [35]. The use of traditional herbal medicines to prevent and treat a variety of diseases has generated considerable interest. Traditionally, SGJT has been used to improve spleen and stomach function, which plays a central role in the health and vitality of the body. According to Traditional Chinese Medicine, menopausal symptoms are associated with a decline in spleen or stomach energy. Therefore, we evaluated the therapeutic effects of SGJT on lipid related diseases in a rat model of menopausal hyperlipidemia.

First, we performed the quantitative analysis of liquiritin and glycyrrhizin in SGJT using a high-performance liquid chromatography (HPLC). Identifying the major components is very important because their origin is relevant to the effects of the herbal medicine. Then, we explored the effects of SGJT on a number of targets associated with lipid related diseases, including retroperitoneal fat, perirenal fat, serum lipid levels, the atherogenic index, cardiac risk factors, lumen diameter, media thickness, and NASH, in a rat model of menopausal hyperlipidemia. Rats were ovariectomized and fed a diet rich in fats or cholesterol, followed by treatment with SGJT. SGJT administration decreased retroperitoneal and perirenal fat, serum TC, TG, and LDL levels, the atherogenic index, cardiac risk factors, and the intima-media thickness. Moreover, SGJT was shown to ameliorate NASH and increase the lumen diameter and HDL levels to those similar to the positive controls. These results show that SGJT can improve symptoms caused by menopausal hyperlipidemia.

Some natural products are used to manage metabolic syndrome during menopause. For example,* Nigella sativa* showed therapeutic and protective effects against metabolic syndrome by modifying weight gain and improving the lipid profile and blood glucose and hormone levels in ovariectomized rats [36]. Flaxseed reduced plasma cholesterol levels and atherosclerotic lesion formation induced by ovarian hormone deficiency in hamsters [37]. Like these reports, SGJT has therapeutic and protective effect against metabolic syndrome during menopause. Since SGJT has effects on not only one symptom but also multiple targets associated with lipid related diseases, SGJT might be more useful than other existing natural products for the treatment of lipid related diseases in menopausal rat.

In the clinical setting, some studies have reported a relationship between the intake of natural products and menopausal symptoms. Flaxseed taken at a dose ranging from 40 to 50 g/day was also shown to have cholesterol-lowering properties in postmenopausal women [38, 39]. An isoflavone containing genistein, daidzein, formononetin, and biochanin extracted from red clover increased HDL and decreased apolipoprotein B levels when taken at doses of 28.5, 57, or 85.5 mg/day in postmenopausal women [40]. Isoflavone (1 : 1 : 0.2 genistein : daidzein : glycitein) taken at 90 mg/day improved vascular reactivity in postmenopausal women with hypercholesterolemia [41]. Dehydroepiandrosterone at a dose of 25 mg/day showed improved lipid patterns [42]. Whether SGJT could improve lipid related disease in postmenopausal females will be a subject in our future research plan.

Additionally, we carried out an experiment in the M*β*CD-induced hepatic steatosis model in HepG2 cell to investigate the cholesterol-lowering effect of SGJT. We showed that M*β*CD treatment alone caused a significant increase in lipid accumulation and TC and LDL/VLDL levels, all of which were reduced following treatment with SGJT (Figure 4). Together, these results show that SGJT exerts cholesterol-lowering effects on HepG2 cells.

Cholesterol is an essential molecule for maintaining membrane structure and is a precursor of steroid hormones, bile acids, and vitamin D [43]. Cholesterol, whether obtained from the diet or synthesized* de novo*, is transported through the circulation in small lipoprotein particles. Intracellular cholesterol levels are maintained by a tightly regulated feedback system that controls the biosynthesis, influx, catabolism, and efflux of cholesterol [17, 44]. Failure to properly regulate cholesterol levels leads to the abnormal deposition of cholesterol and cholesterol-rich lipoproteins, resulting in a wide range of diseases including hyperlipidemia, cirrhosis, fatty liver disease, cardiovascular disease, diabetes, and atherosclerosis.

The primary regulator of cholesterol metabolism is SREBP2, which activates the expression of genes required for cholesterol biosynthesis, including HMGCS, HMGCR, LDLR, farnesyl diphosphate synthase, and squalene synthase [19]. Generally speaking, a decrease in intracellular cholesterol triggers SREBP2 activation, which in turn activates both HMGCR and LDLR and leads to an increase in intracellular cholesterol concentrations [44]. In contrast, an increase in intracellular cholesterol leads to the downregulation of SREBP2 and a decrease in intracellular cholesterol concentrations. M*β*CD treatment alone led to increased cholesterol levels and subsequent downregulation of the effector proteins SREBP2, LDLR, and HMGCR (Figure 5). Cotreatment with SGJT and M*β*CD decreased cholesterol levels, resulting in increased expression of SREBP2 and LDLR (Figure 5). There are some reports that the upregulation of either SREBP2 or LDLR is responsible for improved cholesterol levels. For example, an astaxanthin-rich extract from the green alga* Haematococcus pluvialis* exhibits a hypocholesterolemic effect through the upregulation of LDLR expression [45]. Resveratrol increases the expression and activity of LDLR in hepatocytes via activation of SREBPs and exhibits antiatherogenic effects [46]. Resveratrol protected against the high-fat/sucrose diet-induced decrease in hepatic LDLR [47]. However, in contrast with the normal regulatory response, the expression of HMGCR was decreased (Figure 5). In these experiments, we used simvastatin as a positive control, as this drug is known to suppress HMGCR activity and, therefore, reduce intracellular cholesterol levels [48]. The data presented here suggest that the response to SGJT was similar to that of simvastatin in terms of decreasing cholesterol synthesis in HepG2 cells exposed to M*β*CD.

Increased AMPK phosphorylation was also observed following SGJT treatment (Figure 6). AMPK acts as a central regulator of lipid metabolism [49], governing lipid homeostasis via alternative activation of catabolic and anabolic pathways [21, 49, 50]. Based on its role as a key regulator of lipid homeostasis, AMPK has emerged as a promising target in the treatment of fatty liver disease. Certain natural products including* Artemisia sacrorum* Ledeb., luteolin, mulberry extract, and curcumin attenuate hepatic lipid accumulation via AMPK activation [30, 49, 51, 52]. Thus, SGJT might also regulate cholesterol synthesis via AMPK phosphorylation. Overall, present data* in vitro* suggest that inhibition of lipid synthesis on M*β*CD-induced HepG2 cells by SGJT blocks the progression of hepatocyte steatosis.

We believe SGJT is a novel combination medicine with health-promoting benefits that can improve multiple lipid-associated factors in menopause.

## 5. Conclusions

In conclusion, we have shown that SGJT may be used as a novel agent to treat or prevent high-cholesterol and high-fat-induced lipid related disease during menopause. Our results also support the view that the antisteatosis effects of SGJT may be attributed to regulation of cholesterol synthesis pathway and activation of AMPK.

## Figures and Tables

**Figure 1:** Chromatograms of SGJT aqueous extract and 2 reference standards of glycyrrhizin (254 nm) and liquiritin (280 nm).

**Figure 2:** Histological analysis of adipose tissue and livers in a rat model of menopausal hyperlipidemia. Sham: Sham rats fed a high-fat (HFD), high-cholesterol diet (HCD); Con: OVX rats fed a high-fat (HFD), high-cholesterol diet (HCD); SV: OVX rats fed a high-fat (HFD), high-cholesterol diet (HCD) supplemented with simvastatin (20 mg/kg); SG-50: OVX rats fed a high-fat (HFD), high- cholesterol diet (HCD) supplemented with SGJT (50 mg/kg); SG-150: OVX rats fed a high-fat (HFD), high-cholesterol diet (HCD) supplemented with SGJT (150 mg/kg). After 8 weeks, adipose tissues (a) and livers (b) were extracted and stained with H&E (adipose tissues: ×100 magnification, livers: ×400 magnification).

**Figure 3:** Cytotoxicity of M*β*CD and SGJT in HepG2 cells. HepG2 cells were treated with several concentrations of SGJT (250–1,000 *μ*g/mL) for 8 h in 0.2% BSA-DMEM, and the cell viability was determined using WST assay (a). HepG2 cells were treated with 20 mg/mL M*β*CD and 30 *μ*M simvastatin or several concentrations of SGJT (250–1,000 *μ*g/mL) with 20 mg/mL M*β*CD for 8 h in 0.2% BSA-DMEM, and the cell viability was determined using WST assay (b). The data were mean ± SD from three samples for each group. Values not sharing a common alphabet as superscripts are significantly different from each other at the level of *P* < 0.05 (ANOVA followed by Duncan's test). Similar results were obtained in three separate experiments.

**Figure 4:** Effects of SGJT on lipid accumulation, total cholesterol, and LDL/VLD levels in HepG2 cells. HepG2 cells were treated with 30 *μ*M simvastatin or several concentrations of SGJT (250–1,000 *μ*g/mL) with 20 mg/mL M*β*CD for 8 h in 0.2% BSA-DMEM. Lipid accumulation was visualized by Oil Red O staining (×600 magnification) and quantitative analysis of lipid deposition in cells was analyzed by spectrophotometer (a). Total intracellular cholesterol (b) and LDL/VLDL (c) levels were measured by ELISA. The data were mean ± SD from three samples for each group. ^##^Significantly different between the control and M*β*CD treatment at *P* < 0.01 (two-sample *t*-test). Values not sharing a common alphabet as superscripts are significantly different from each other at the level of *P* < 0.05 (ANOVA followed by Duncan's test). Similar results were obtained in three separate experiments.

**Figure 5:** Effects of SGJT on cholesterol synthesis in HepG2 cells. HepG2 cells were treated with 30 *μ*M simvastatin or SGJT (250, 500 *μ*g/mL) with 20 mg/mL M*β*CD for 8 h in 0.2% BSA-DMEM. Cell lysates were then harvested by RIPA buffer and subjected to HMG-CoA reductase activity and inhibition assays (a) and Western blotting analysis for SREBP2, HMGCR, and LDLR protein expression (b). Quantified data of protein levels indicated in lower panel. The values of density of proteins were all justified with *β*-actin. The relative density ratios of untreated cells were set at a value of 1.0. Values not sharing a common alphabet as superscripts are significantly different from each other at the level of *P* < 0.05 (ANOVA followed by Duncan's test). Similar results were obtained in three separate experiments.

**Figure 6:** Effects of SGJT on AMPK phosphorylation in HepG2 cells. HepG2 cells were treated with 30 *μ*M simvastatin or SGJT (250, 500 *μ*g/mL) with 20 mg/mL M*β*CD for 8 h in 0.2% BSA-DMEM. Cell lysates were then harvested and subjected to Western blotting analysis for AMPK phosphorylation (pThr-172-AMPK). Quantified data of protein levels indicated in lower panel. The values of density of proteins were all justified with *β*-actin. The relative density ratios of untreated cells were set at a value of 1.0. Values not sharing a common alphabet as superscripts are significantly different from each other at the level of *P* < 0.05 (ANOVA followed by Duncan's test). Similar results were obtained in three separate experiments.

**Table 1:** Metabolic parameters in a rat model of menopausal hyperlipidemia.

	Sham	OVX-Con	OVX-SV	OVX-SGJT (50)	OVX-SGJT (150)	OVX-SGJT (450)
	(*n* = 5)	(*n* = 5)	(*n* = 5)	(*n* = 5)	(*n* = 5)	(*n* = 5)
Body weight gain (g)	96.44 ± 4.8	117.34 ± 1.9^a∗^	85.74 ± 3.0^d^	109.40 ± 2.3^b^	92.12 ± 2.5^c^	96.02 ± 2.7^c^
Food intake (g/day)	57.60 ± 18.90^a^	58.65 ± 18.75^a^	53.30 ± 14.40^a^	54.25 ± 14.95^a^	53.85 ± 15.15^a^	55.20 ± 15.70^a^
Liver weight (g)	7.673 ± 0.413	17.510 ± 1.351^a∗^	15.609 ± 1.043^a^	16.080 ± 1.467^a^	17.361 ± 1.032^a^	17.598 ± 1.094^a^
Retroperitoneal fat (mm)	119.03 ± 8.56	217.96 ± 18.08^a∗^	108.02 ± 6.81^b^	86.11 ± 4.45^b^	95.08 ± 6.85^b^	95.99 ± 4.52^b^
Perirenal fat (mm)	89.4355 ± 1.67	233.87 ± 10.10^a∗^	100.37 ± 11.64^b^	81.45 ± 6.63^b^	84.99 ± 5.49^b^	94.85 ± 3.37^b^

Sham, Sham rats fed a high-fat (HFD), high-cholesterol diet (HCD); OVX-Con, OVX rats fed a high-fat (HFD), high-cholesterol diet (HCD); OVX-SV, OVX rats fed a high-fat (HFD), high-cholesterol diet (HCD) supplemented with simvastatin (20 mg/kg); OVX-SGJT, OVX rats fed a high-fat (HFD), high-cholesterol diet (HCD) supplemented with SGJT (50, 150, 450 mg/kg). After 8 weeks, body, and liver weights (g) and retroperitoneal fat and peri-renal fat sizes (mm) were measured. Values are expressed as means ± SD (*n* = 5). ^∗^Significantly different between the sham and OVX-Con at *P* < 0.01, (two-sample *t*-test). Values not sharing a common alphabet as superscripts are significantly different from each other at the level of *P* < 0.05 (ANOVA followed by Duncan's test).

**Table 2:** Serum lipid levels in a rat model of menopausal hyperlipidemia.

	Sham	OVX-Con	OVX-SV	OVX-SGJT (50)	OVX-SGJT (150)	OVX-SGJT (450)
	(*n* = 5)	(*n* = 5)	(*n* = 5)	(*n* = 5)	(*n* = 5)	(*n* = 5)
T-CHO (mg/dL)	113.50 ± 2.179	221.25 ± 6.142^a∗∗^	178.50 ± 35.624^bc^	147.00 ± 3.894^c^	178.75 ± 0.081^bc^	195.75 ± 18.6221^ab^
TG (mg/dL)	46.6 ± 7.80	64.06 ± 6.06^a∗^	48.33 ± 3.21^a^	46.25 ± 4.66^a^	60.00 ± 4.38^a^	56.75 ± 10.56^a^
HDL (mg/dL)	67.2 ± 4.03	31.8 ± 4.5^a∗∗^	41.6 ± 3.14^b^	36.00 ± 2.71^ab^	41.8 ± 8.31^b^	44.00 ± 3.86^b^
LDL (mg/dL)	37.52 ± 3.83	176.64 ± 0.43^a∗∗^	127.23 ± 31.842^bc^	101.89 ± 3.879^c^	125.08 ± 17.947^bc^	151.75 ± 15.823^ab^

Sham, Sham rats fed a high-fat (HFD), high-cholesterol diet (HCD); OVX-Con, OVX rats fed a high-fat (HFD), high-cholesterol diet (HCD); OVX-SV, OVX rats fed a high-fat (HFD), high-cholesterol diet (HCD) supplemented with simvastatin (20 mg/kg); OVX-SGJT, OVX rats fed a high-fat (HFD), high-cholesterol diet (HCD) supplemented with SGJT (50, 150, 450 mg/kg). After 8 weeks, the serum levels of TC, TG, HDL, and LDL were measured. Values are expressed as means ± SD (*n* = 5). ^∗^Significantly different between the sham and OVX-Con at *P* < 0.01, ^∗∗^ *P* < 0.001 (two-sample *t*-test). Values not sharing a common alphabet as superscripts are significantly different from each other at the level of *P* < 0.05 (ANOVA followed by Duncan's test).

**Table 3:** Atherogenic index, cardiac risk factor, lumen diameter, and media thickness in a rat model of menopausal hyperlipidemia.

	Sham	OVX-Con	OVX-SV	OVX-SGJT (50)	OVX-SGJT (150)	OVX-SGJT (450)
	(*n* = 5)	(*n* = 5)	(*n* = 5)	(*n* = 5)	(*n* = 5)	(*n* = 5)
Atherogenic index	0.69 ± 0.09	6.05 ± 0.89^a∗^	3.31 ± 0.80^b^	3.10 ± 0.284^b^	3.39 ± 0.884^b^	3.47 ± 0.503^b^
Cardiac risk factor	1.69 ± 0.09	7.05 ± 0.89^a∗^	4.31 ± 0.80^b^	4.1 ± 0.284^b^	4.39 ± 0.885^b^	4.47 ± 0.503^b^
Lumen diameter (*μ*m)	1,931.25 ± 2.86	847.78 ± 55.50^a∗∗^	885.39 ± 74.43^ab^	1,000.65 ± 83.5^bc^	974.43 ± 47.84^abc^	1,064.38 ± 81.55^c^
Intima-media thickness (*μ*m)	97.65 ± 12.65	217.66 ± 24.01^a∗^	118.62 ± 11.93^b^	121.44 ± 11.71^b^	109.43 ± 9.41^b^	114.61 ± 10.10^b^
Lumen diameter/intima-media thickness	20.00 ± 2.26	3.75 ± 0.16^a∗^	7.51 ± 0.86^b^	8.29 ± 0.92^bc^	8.95 ± 0.77^bc^	9.34 ± 0.95^c^

Sham, Sham rats fed a high-fat (HFD), high-cholesterol diet (HCD); OVX-Con, OVX rats fed a high-fat (HFD), high-cholesterol diet (HCD); OVX-SV, OVX rats fed a high-fat (HFD), high-cholesterol diet (HCD) supplemented with simvastatin (20 mg/kg); OVX-SGJT, OVX rats fed a high-fat (HFD), high-cholesterol diet (HCD) supplemented with SGJT (50, 150, 450 mg/kg). After 8 weeks, their serum lipid levels were measured, followed by calculation of atherogenic index and cardiac risk factor scores (atherogenic index = (TC − HDL)/HDL, cardiac risk factor = TC/HDL). And lumen diameter and intima-media thickness were measured. Values are expressed as means ± SD (*n* = 5). ^∗^Significantly different between the sham and OVX-Con at *P* < 0.01, ^∗∗^ *P* < 0.001 (two-sample *t*-test). Values not sharing a common alphabet as superscripts are significantly different from each other at the level of *P* < 0.05 (ANOVA followed by Duncan's test).

**Table 4:** NASH scores in a rat model of menopausal hyperlipidemia.

	Sham	OVX-Con	OVX-SV	OVX-SGJT (50)	OVX-SGJT (150)	OVX-SGJT (450)
	(*n* = 5)	(*n* = 5)	(*n* = 5)	(*n* = 5)	(*n* = 5)	(*n* = 5)
Steatosis	0.20 ± 0.20	2.50 ± 0.20^a∗∗^	1.20 ± 0.20^c^	1.00 ± 0.20^c^	0.80 ± 0.20^c^	1.80 ± 0.37^b^
Lobular inflammation	1.00 ± 0.00	2.40 ± 0.24^a∗^	1.40 ± 0.24^b^	1.20 ± 0.20^b^	1.00 ± 0.45^b^	1.40 ± 0.24^b^
Hepatocellular ballooning	1.00 ± 0.00	2.30 ± 0.20^a∗^	1.00 ± 0.00^d^	1.40 ± 0.24^c^	0.40 ± 0.24^e^	1.80 ± 0.20^b^

Sham, Sham rats fed a high-fat (HFD), high-cholesterol diet (HCD); OVX-Con, OVX rats fed a high-fat (HFD), high-cholesterol diet (HCD); OVX-SV, OVX rats fed a high-fat (HFD), high-cholesterol diet (HCD) supplemented with simvastatin (20 mg/kg); OVX-SGJT, OVX rats fed a high-fat (HFD), high-cholesterol diet (HCD) supplemented with SGJT (50, 150, 450 mg/kg). After 8 weeks, steatosis, and lobular inflammation and hepatocellular ballooning contents were measured. Total scores of each component were then added to determine the presence or absence of NASH, with score ≥5 diagnosed as NASH, and scores ≤2 defined as not NASH. Values are expressed as means ± SD (*n* = 5). ^∗^Significantly different between the sham and OVX-Con at *P* < 0.01, ^∗∗^ *P* < 0.001 (two-sample *t*-test). Values not sharing a common alphabet as superscripts are significantly different from each other at the level of *P* < 0.05 (ANOVA followed by Duncan's test).
